RETRACTED

# The Anatase Phase of Nanotopography Titania with Higher Roughness Has Better Biocompatibility in Osteoblast Cell Morphology and Proliferation

**DOI:** 10.1155/2020/8032718

**Published:** 2020-09-22

**Authors:** Danping Ruan, Chunyun Wu, Sinan Deng, Yu Zhang, Guoling Guan

**Affiliations:** Minhang Branch, Zhongshan Hospital, Fudan University, China

## Abstract

Previous studies have concluded that surface-modified titanium oxide (titania, TiO_2_) surface properties promote osteoblast cell morphology and proliferation. To screen a suitable structured titania coating with the best biocompatibility to be used in dental implants, five titania films (two amorphous, one rutile, and two anatases) with different surfaces were successfully synthesized on polished titanium by radio frequency (RF) magnetron sputtering. We applied atomic force microscopy (AFM) and X-ray diffraction (XRD) to depict the formulations. Furthermore, MC3T3-E1, the mouse osteoblast precursor cell, was used to assess cell proliferation and observe morphologic changes at the film surface. The data indicated that the overall number of MC3T3-E1 cells on anatase films was significantly higher as compared with cells on rutile and amorphous films. Meanwhile, the actin filaments of the cells grown on the anatase phase films were well defined and fully spread. In addition, the film with higher roughness had enhanced biocompatibility than that with lower roughness. The results showed that the crystal phase and titania coated roughness had a greater influence on the biocompatibility of nanostructured titania film. The higher the roughness of the anatase phase was, the better bioactivity for the morphology and proliferation of osteoblast. This is a good surface-modified biological material and may have a good application prospect in dental implants.

## 1. Introduction

The wide application of titanium (Ti) and its alloys as implants in oral implantology is due to such advantages as light mass, high specific strength, resistance to corrosion, low modulus of elasticity, and biocompatibility [1]. Although the success rate of titanium implants is high, 5%-10% of these implants still fails [2, 3], mostly because of failed biocompatibility of the implants [4, 5], which are influenced by surface properties of the implant [6–9]. It was reported that surface energy and wettability were two key factors that stimulated osteoblast response leading to osseointegration between bone and implant [10]. Moreover, the surface roughness of implant is also conducive to osteoblast differentiation. It is well known that the rough and porous surface structure can promote osteoblast migration and growth into the porous surface through enlarging the contact area between the implant material and its surrounding osteoblasts [11].

RETRACTED

Based on the understanding of natural bone, the modification of the surface properties of Ti implants at the nanoscale level is the best way to improve its biocompatibility, which mimics the properties of human bone surface and alleviates the stimulation of the surrounding environment [12–14]. Studies on thin-film coating of implant surfaces have been conducted by many researchers using different approaches, and the thin-film coating has been widely used in the clinic [15–19]. However, some defects, such as phase changes leading to poor adhesion, nonuniformity, and microcrack formation, limit the application of these methods in implant systems [20, 21]. Magnetron sputtering deposition is a flexible technique, which is recently developed, and it also has many advantages including ease of sputtering any material, high deposition rates, extremely high adhesion to films, the formation of high-purity films, and dense coatings. Thus, it is widely used in the surface modification of implants. Using this technique, many groups successfully synthesized the crystal phase of titania on the surface of biomaterials [22] and the different crystal phases of nanotopography titania had diverse biocompatibility for osteoblast responses and osseointegration [23].

In our study, we deposited 5 titania films with different crystal phases and roughness on Ti substrates by RF magnetron sputtering. Furthermore, the mouse osteoblast precursor cell MC3T3-E1 was used to investigate cell responses to the different titania films.

## 2. Material and Methods

### 2.1. Fabrication of Nanostructured Titania Films

RF magnetron sputtering system (JGP-450 A, SKY Technology Development Co., Ltd, CAS, China) was applied to deposit the titania films according to previously reported methods [1], and its corresponding principle is shown in Figure 1. Finally, five kinds of specimens were fabricated and Table 1 presents the deposition conditions.

### 2.2. Surface Characterization

Deposited on Ti substrates at different working pressures with RF power of 150 W, the phase characterization of the titania films with or without bias was conducted by Powder Diffraction File (XRD PDF-2 2018) and the surface topography of the titania films was featured by atomic force microscopy (AFM, Nanoscope 3A, DI, USA) [24]. The roughness of root-mean-square (RMS) was assessed by Nanoscope® III [1].

### 2.3. Cell Culture

The MC3T3-E1 cells were purchased from American Type Culture (ATCC, Manassas, VA, USA) and cultured in a proliferation medium containing *α*MEM (Gibco, Paisley, UK) added with 10% fetal bovine serum (Gibco, Grand Island, NY) and 100 units/ml penicillin/streptomycin in a humidified incubator set at 37°C and 5% CO_2_. Then, cells were digested using trypsin/EDTA (Hyclone, Bonn, Germany) and resuspended in the supplemented culture medium. Subsequently, the cells were seeded on the specimen surfaces for further research, and every square centimeter was seeded 2 × 10^4^ cells.

RETRACTED

### 2.4. Cell Proliferation Assay

Cells were fixed with 4% paraformaldehyde (PFA, Sigma, USA) for 30 min and then the fixed cells were stained with 4′,6-diamidino-2-phenylindole (DAPI, Sigma, USA). Cells were examined with a fluorescent microscope (200x), and the number of cells was estimated by the ImageJ software for at least five random observation fields of each specimen.

### 2.5. Actin Cytoskeleton Assay

After growing on the specimen surfaces for 12 h, the cells were rinsed with PBS. The collected cells were processed for the following steps: fixed in 4% PFA for 20 min, washed in PBS, permeabilized with 0.1% Triton X-100 for 4 min, and washed in PBS again. To avoid nonspecific background staining, 3% bovine serum albumin was applied to block the cells, and then, the cells were stained for 20 min by fluorescent rhodamine phalloidin (Invitrogen, USA). After being washed in 0.01 mol/l PBS, the specimens were fixed onto coverslips using cytospin (Thermo, USA) and sealed with Mounten Media (Invitrogen, USA). The actin cytoskeleton was examined through a confocal laser scanning microscope (CLSM, TCS SP2, Leica, Germany) which was adapted for the inverted microscope. Finally, a 200x (NA 1.4, oil) Leitz Plan-Apochromatic objective was used to take the images.

### 2.6. Statistical Analysis

Data were expressed as the mean ± SD, and differences between groups were analyzed using the SPSS software 20.0 (SPSS Inc., Chicago, IL, USA). Each experiment was repeated no less than three times. Student's *t*-test was conducted to examine the significance of results. A *P* value less than 0.05 was thought to be significant.

## 3. Results

### 3.1. Structural Characterization

To screen a suitable structured titania coating with the best biocompatibility in dental implants, we generated five types of specimens. Briefly, with the same deposition power (*P* = 150 W), different working pressures (*P* = 3, 5, and 7 Pa) and substrate bias (0 and 50 V) were utilized to get different types of crystal phase titania. The acquired specimens were named T3P0V, T5P0V, T7P0V, T5P50V, and T7P50V according to the working pressures and substrate bias.

The XRD results in Figure 2 showed that when the total pressure was 3 or 5 Pa and the substrate bias was 0 V, no diffraction peaks were detected in T3P0V (Figure 2(a)) and T5P0V (Figure 2(b)) films. Thus, the T3P0V and T5P0V films were either containing ultrasmall nanocrystallites undetectable by XRD or purely amorphous. When the pressure was added to 7 Pa, stable rutile was clearly observed in the oxide coatings of T7P0V (Figure 2(c)). Meanwhile, at the 50 V substrate bias, the T5P50V (Figure 2(d)) and T7P50V (Figure 2(e)) diffraction patterns indicated that the T5P50V and T7P50V films were composed of anatase titania.

RETRACTED

The AFM results in Figure 3 showed the 3D surface morphology of the titania film. The surface roughness was measured: 16.27 nm for T3P0V, 8.529 nm for T5P0V, 16.75 nm for T7P0V, 20.48 nm for T5P50V, and 40.51 nm for T7P50V. The T5P0V film had the lowest surface roughness, and the T7P50V film had the highest surface roughness. Although T3P0V and T7P0V showed different crystal phases, they had similar surface roughness. Meanwhile, T5P50V and T7P50V showed the same crystal phases, but T7P50V had higher surface roughness.

The crystal phase and roughness of five films are shown in Table 2.

### 3.2. Cell Proliferation on Titania Samples

Images of cell growth on the five specimen surfaces are shown in Figure 4. It was demonstrated that all types of specimen surfaces were suitable for MC3T3-E1 cell growth. However, significant differences were found. The cell number in the T7P50V group was the highest in five groups (*P* < 0.05), the T5P50V group came second, and the T7P0V group came third. The T3P0V and T5P0V groups were the lowest, although the T3P0V group seemed higher than the T5P0V group (*P* > 0.05).

### 3.3. Cytoskeleton

After growing on the specimen surface for 12 h, MC3T3-E1 cells were stained by rhodamine phalloidin and the cytoskeleton images were taken by a confocal microscope and shown in Figure 5. According to the morphology, the cells that are attached on the surface of the specimen can be divided into three types [25]. Firstly, not spread type is that cells are still spherical, and protrusions are not yet produced. Secondly, partially spread type is that cells start to spread laterally at one or more sides. Thirdly, fully spread type is cells that at this stage the extensions of plasma membrane are completely confluent. The cells in the T3P0V and T5P0V groups were either spherical or spread laterally at one or more sides (Figures 5(a) and 5(b)). Although the cells in the T7P0V and T5P50V groups were completely spread, the actin filaments extended in irregular directions (Figures 5(c) and 5(d)). The actin filament distribution was fully spread in the T7P50V group (Figure 5(e)). Moreover, all of the actin filaments with regular directions in the T7P50V group were well defined and the actin microfilament system was parallel with the long axis of the cells.

RETRACTED

## 4. Discussion

Over the past decades, titanium and its alloys have been widely applied as biomaterials in the field of implants, because of their appropriate properties, such as good biocompatibility and mechanical characteristics, corrosion resistance, and process ability [26]. However, as a kind of bioinert material, pure titanium shows bad osteoblast responses and osseointegration with bone tissue. It has been proved that the interactions between the surface of biomaterials and the biological environment depend on the surface of implants [27, 28]. It is well known that cellular responses are determined by a biomaterial surface's physical structure. Therefore, to acquire appropriate properties for biomedical applications, surface modification is broadly applied [29]. With the development of material chemistry, it is demonstrated that the nanoscale features, particularly the crystal phase, significantly influence cell behavior [30]. In the previous study, different crystal phases of titania film have been synthesized and it is widely considered that the anatase phase of titania is a core factor on osteoblast cell morphology and proliferation [23]. The purpose of this study is to acquire a greater depth of understanding of the subject and put forward a new proposal for surface modification and suitable biomaterial to be used in dental implants.

In our study, we successfully synthesized five titania films (one rutile, two anatases, and two amorphous titania) of different roughness on polished titanium by RF magnetron sputtering. We found that the cell morphology and bone architecture of MC3T3-E1 cells on five titania film surfaces were greatly diverse. In the T7P50V group, the distribution of actin filament was evenly spread and the actin microfilament system was parallel with the long axis of the cells, which might be affected by the nanotopography [31]. It is well known that spreading is a key step in cell adhesion, which has great potential for contributing to cell proliferation [32, 33]. In this study, cell proliferation was also increased in the T7P50V group (anatase phase with higher roughness), which led to a faster and distinct polygonal spreading of the cells.

In sum, we deeply investigated the role of the crystal phase and roughness of nanotopography titania in osteoblast cell morphology and proliferation. From the crystal phase standpoint, our results showed that the anatase phase (T5P50V and T7P50V) had the best biocompatibility, the rutile phase (T7P0V) came second, and amorphous titania (T3P0V and T5P0V) came third. Meanwhile, from the roughness standpoint, the results showed that the films with higher roughness (T7P50V>T5P50V>T7P0V>T3P0V>T5P0V) had higher biocompatibility. Based on the results above, T7P50V is a suitable structured titania coating with the best biocompatibility that can be used in dental implants.

RETRACTED

## 5. Conclusions

Our results indicate that the roughness and configuration of the surface of implant materials may modulate the spreading and proliferation of their surrounding cells. Cells spread and grow better on the anatase phase with higher roughness, which may provide a potential measure for the surface modification of dental implants.

## Figures and Tables

**Figure 1:** Schematic diagram of RF magnetron sputtering.

**Figure 2:** XRD patterns of (a) T3P0V, (b) T5P0V, (c) T7P0V, (d) T5P50V, and (e) T7P50V.

**Figure 3:** AFM pictures of titanium dioxide layer deposition by RF magnetron sputtering: (a) T3P0V, (b) T5P0V, (c) T7P0V, (d) T5P50V, and (e) T7P50V.

**Figure 4:** Images of MC3T3-E1 cells grown on (a) T3P0V, (b) T5P0V, (c) T7P0V, (d) T5P50V, and (e) T7P50V surfaces. (f) Proliferation of MC3T3-E1 cells. ^∗^*P* < 0.05 compared with the other four groups. ^#^*P* < 0.05 compared with the other three groups.

**Figure 5:** Images of MC3T3-E1 cells spread on (a) T3P0V, (b) T5P0V, (c) T7P0V, (d) T5P50V, and (e) T7P50V surfaces.

**Table 1:** Summary of deposition conditions of titania films.

Base pressure	1.4 × 10^−3^ Pa
Working pressures	T3P0V: 3 Pa at a substrate bias of 0 V
	T5P0V: 5 Pa at a substrate bias of 0 V
	T7P0V: 7 Pa at a substrate bias of 0 V
	T5P50V: 5 Pa at a substrate bias of 50 V
	T7P50V: 7 Pa at a substrate bias of 50 V
Deposition time	8 hrs for each sample
RF power	150 W
Argon flow rate	30 sccm
Oxygen flow rate	10 sccm
Target to substrate distance	70 mm
Diameter of silicon (100) substrate	25.4 mm
Diameter of the titanium target	60 mm

**Table 2:** Summary of crystal phase and roughness of titania films.

Film	Crystal phase	Roughness
T3P0V	Amorphous	16.27 nm
T5P0V	Amorphous	8.529 nm
T7P0V	Rutile	16.75 nm
T5P50V	Anatase	20.48 nm
T7P50V	Anatase	40.51 nm

## Data Availability

All data generated or analyzed during this study are included in this published article.
